# Survival and clinicopathological characteristics of cT4b oral squamous cell carcinoma based on different treatment modalities: A single-center retrospective study

**DOI:** 10.1097/MD.0000000000029285

**Published:** 2022-05-20

**Authors:** Nan-Chin Lin, Jui-Ting Hsu, Michael Y.C. Chen, Kuo-Yang Tsai

**Affiliations:** a School of Dentistry, China Medical University, Taichung, Taiwan; b Department of Oral and Maxillofacial Surgery, Show Chwan Memorial Hospital, Changhua, Taiwan; c Department of Bioinformatics and Medical Engineering, Asia University, Taichung, Taiwan; d Department of Oral and Maxillofacial Surgery, China Medical University Hospital, Taichung, Taiwan.

**Keywords:** oral cavity cancer, oral squamous cell carcinoma, surgical treatment, T4b

## Abstract

**Introduction:**

Primary surgical treatment for oral squamous cell carcinoma (OSCC) is reserved for T1 to T4a tumors, but not for T4b tumors, according to the present National Comprehensive Cancer Network clinical practice guidelines. In this retrospective study, we aimed to determine the association between the clinicopathological characteristics and different treatment modalities for T4b OSCC based on whether patients received primary surgical treatment. Therefore, we conducted a survival analysis based on different treatment modalities.

**Methods:**

This retrospective cohort study enrolled 125 patients with clinical stage T4b OSCC who received treatment and were followed up at Changhua Christian Hospital between January 1, 2008 and December 31, 2018.

**Results:**

Overall, 81 patients received primary surgical treatment and 44 received primary nonsurgical treatment. Comparison of the clinicopathological characteristics between those who did and did not undergo surgery revealed no significant differences in age at tumor diagnosis, tumor location, clinical N stage, and involved tumor area based on computed tomography or magnetic resonance imaging, or stratified Charlson Comorbidity Index scores. In the survival analysis, Kaplan–Meier curves revealed that patients who received treatment modalities including surgery exhibited better survival than those who received treatment modalities that did not include surgery.

**Conclusions:**

In the present study, patients with T4b OSCC treated with primary surgery had a better overall survival rate than those who received nonsurgical treatment. In the future, it will be necessary for clinicians worldwide to report the treatment outcomes of patients with T4b OSCC based on the common criteria.

## 1 Introduction

Oral squamous cell carcinomas (OSCCs) that involve the masticator space, pterygoid plates, or skull base, or that encase the internal carotid artery, are classified as T4b, according to the American Joint Committee on Cancer (AJCC) staging system.^[1]^ Primary surgical treatment for OSCC is reserved for T1 to T4a tumors, but not for T4b tumors, according to the present National Comprehensive Cancer Network (NCCN) clinical practice guidelines.^[2]^ Moreover, limited reports of treatment outcomes of T4b OSCC patients have been published. One reason why surgery is not performed in patients with T4b tumors may be that T4b OSCC tumors involve the masticator space, which increases the difficulty of radical resection. Additionally, T4b OSCC patients have a relatively poor prognosis, and the NCCN clinical practice guidelines have proposed treatment with palliative intent or clinical trials for those patients. Hence, heterogeneous treatment protocols have also been reported.^[3–7]^

In the present retrospective study, we aimed to determine the association between the clinicopathological characteristics and different treatment modalities for T4b OSCC based on whether patients received primary surgical treatment or some other treatment. To accomplish this, we conducted a survival analysis based on different treatment modalities.

## 2 Methods

### 2.1 Patients

This retrospective cohort study was approved by the Institutional Review Board and Ethics Committee of Changhua Christian Hospital (IRB No. 210210). All clinical data were obtained through chart review and from the cancer registry center. A total of 177 patients who were diagnosed with clinical stage T4b oral cavity OSCC were identified; all received treatment and were followed up at Changhua Christian Hospital between January 1, 2008, and December 31, 2018. The follow-up duration began at indexing and ended on June 30, 2019. The exclusion criteria included patients who did not receive any treatment (n = 14), those who were lost to follow-up or had incomplete data (n = 18), those who were initially diagnosed with recurrence or distant metastasis (n = 15), and those who did not receive treatment at Changhua Christian Hospital (n = 5). Finally, 125 patients were identified, included, and subsequently analyzed. Clinical T4b stage was diagnosed by clinical examination and either computed tomography (CT) or magnetic resonance imaging (MRI). Tumors that involve the masticator space and cause trismus, as well as those that involve the pterygoid plates or skull base or that encase the internal carotid artery >270 degree are classified as T4b, according to the AJCC staging system.^[1]^

### 2.2 T4b OSCC treatment protocols

The T4b OSCC patients received surgery enrolled in our study underwent wide tumor excision including mandibulectomy and/or maxillectomy and radical neck dissection. Adjuvant therapy was performed in individual cases by our interdisciplinary head and neck surgery team, which included surgeons, oncology radiologists, a medical oncologist, and a pathologist. In general, induction chemotherapy was administered to patients with TPF (Docetaxel [60 mg/m^2^]/Cisplatin [60 mg/m^2^], and/or not 5-fluorouracil [600 mg/m^2^]) in 1 to 3 cycles and repeated after 3 to 4 weeks. Concurrent radiochemotherapy (CCRT) was performed in all the patients enrolled in our study. Radiotherapy was administered for non-surgery cases or no >6 weeks after surgery and was delivered by a linear accelerator at a total dose of 60 to 66 Gy (1.8–2.0 Gy/fraction). If chemotherapy concurrent with radiotherapy was indicated, cisplatin (80 mg/m^2^) and 5-fluorouracil (400–500 mg/m^2^) were administered in 2 cycles and repeated after 4 to 5 weeks.

### 2.3 Clinical and pathological parameters

The characteristics of patients in all the groups analyzed included age at OSCC diagnosis, survival time, gender, pathological AJCC anatomic site, AJCC TNM stage (7^th^ and 8^th^ editions), diagnostic tools, tumor-involved area based on CT or MRI scan, treatment modalities, and Charlson Comorbidity Index (CCI) scores.^[8]^ The anatomic site can be subclassified into the alveolar ridge, anterior two-thirds of the tongue, buccal mucosa, hard palate, floor of the mouth, retromolar trigone, and mucosa of the lip. Death-related information was obtained from the cancer registry center of Changhua Christian Hospital and from data renewed annually by the Health Bureau of Changhua City. CCI scores were used to evaluate comorbidities in patients to investigate a possible association between treatment modalities and the normal healthy condition of patients. Treatment modalities were subclassified into the following 4 groups: surgery + concurrent chemoradiation therapy (CCRT), induction chemotherapy (IC) + surgery + CCRT, IC + CCRT, and CCRT alone.

Finally, we designed an observational, retrospective study based on the treatment modalities received by patients to compare their clinical and pathological characteristics and to conduct a survival analysis among all the groups.

### 2.4 Statistical analysis

Continuous variables are expressed as means ± standard deviations, whereas categorical variables are expressed as percentages. The *χ*^2^ test was employed to compare the differences in the categorical variables among all the groups. Estimates of the overall survival (OS) rates were calculated *via* Kaplan–Meier analyses. The group survival functions were compared using log-rank tests based on the OS. A *P* value <.05 was considered statistically significant. In multivariate analysis, the Cox proportional hazard model was established to evaluate the significance between clinicopathological factors of tumors and OS of patients. The *χ*^2^ statistic tested the relationship between time and all the covariates in the model and checked the fitness of the model. All statistical analyses were conducted using the statistical package SPSS for Windows (version 16, SPSS, Chicago, IL).

## 3 Results

Overall, 125 patients who were enrolled in our retrospective study were divided into the following two groups: those who received treatment modalities including surgery (case group) and those who received treatment modalities that did not include surgery (control group). Table 1 presents the age, sex, anatomic site of the tumor, clinical N stage, diagnostic tools, tumor-involved area according to CT or MRI, treatment modalities, and CCI scores of all 125 patients. Of all the patients with clinical T4b OSCC, 77 were diagnosed by CT (61.6%), whereas 48 patients were diagnosed by MRI (38.4%). With regard to the tumor-involved area, the masticator space was involved in all patients, the pterygoid plate was involved in 19 patients, 4 patients exhibited tumor invasion into the skull base, and 6 patients demonstrated tumor involvement in the carotid artery. The patients were also divided into 4 groups according to treatment modality: 36 patients received surgery + CCRT (28.8%), 45 patients received IC + surgery + CCRT (36%), 24 patients received IC + CCRT (19.2%), and 20 patients received CCRT alone (16%). Finally, most patients had CCI scores of 2 points (n = 43, 34.4%), whereas 32 (25.6%) and 22 (17.6%) patients had CCI scores of 3 and 5 points, respectively.

**Table 1:** Summary of clinical and pathological data of all patients with T4b OSCC.

	T4b (n = 125)	
	n	%
Age at diagnosis		
≤40	13	10.4
41–50	33	26.4
51–60	49	39.2
61–70	23	18.4
≥71	7	5.6
Gender		
Male	123	98.4
Female	2	1.6
Tumor sites		
Alveolar ridge	30	24.0
Anterior tongue	4	3.2
Buccal mucosa	54	43.2
Hard palate	19	15.2
Floor of mouth	2	1.6
Retromolar trigone	15	12.0
Lip	1	0.8
Clinical N stage		
0	29	23.2
1	11	8.8
2	83	66.4
3	2	1.6
Diagnostic tools		
CT	77	61.6
MRI	48	38.4
Tumor-involved area		
Masticator space	125	
Pterygoid plate	19	
Skull base	4	
Encased ICA	6	
Treatment modalities		
S + CCRT	36	28.8
IC + S + CCRT	45	36.0
IC + CCRT	24	19.2
CCRT only	20	16.0
CCI score		
2	43	34.4
3	32	25.6
4	12	9.6
5	22	17.6
6	9	7.2
7	6	4.8
8	1	0.8

CCI = Charlson Comorbidity Index, CCRT = concurrent chemoradiation therapy, IC = induction chemotherapy, RT = radiotherapy, S = surgery.

As presented in Table 2, 81 patients received primary surgical treatment, and 44 patients received primary nonsurgical treatment. When the clinical and pathological characteristics were compared between the treatment modalities with and without surgery, no significant difference was observed in age at OSCC diagnosis, tumor site, clinical N stage, tumor-involved area based on CT or MRI scan, or stratified CCI scores. CCI scores were used to investigate whether those patients who received primary nonsurgical treatment had a poor comorbid disease status. However, when their survival status was compared (from index date to June 30, 2019), patients who received treatment modalities that included surgery exhibited better survival than those who received treatment modalities without surgery (*P* = .012). All death cases were died from cancer-related mortality including surgery or nonsurgery factors. In nonsurgery group, the major cause of the death was distant metastasis (79.4%), and in the surgery group, the major causes of the death were distant metastasis and local recurrence (both 27.3%). 12 of 81 patients (14.8%) received primary surgical treatment could be achieved in >5 mm surgical margin, and 28 of 81 patients (34.6%) could not achieve enough surgical margin (<1 mm). CCI scores were used to investigate whether those patients who received primary nonsurgical treatment had a poor comorbid disease status.

**Table 2:** Clinical and pathological characteristics of patients treated with different treatment modalities-based primary surgical treatment.

	Treatment modalities including surgery						
	No (n = 44)		Yes (n = 81)		Total (n = 125)		
	n	%	N	%	n	%	*P*
Age at diagnosis							
≤40	3	6.8	10	12.3	13	10.4	.062
41–50	10	22.7	23	28.4	33	26.4	
51–60	14	31.8	35	43.2	49	39.2	
61–70	14	31.8	9	11.1	23	18.4	
≥71	3	6.8	4	4.9	7	5.6	
AJCC anatomic site							
Alveolar ridge	11	25.0	19	23.5	30	24.0	.801
Anterior tongue	1	2.3	3	3.7	4	4.0	
Buccal mucosa	16	36.4	38	46.9	54	54.0	
Hard palate	9	20.5	10	12.3	19	15.2	
Floor of mouth	1	2.3	1	1.2	2	1.6	
RMT	6	13.6	9	11.1	15	12.0	
Mucosa of the lip	0	0.0	1	1.2	1	0.8	
CCI							
<4	23	52.3	52	64.2	75	60.0	.196
≥4	21	47.7	29	35.8	50	40.0	
Tumor-involved area							
Masticator only	37	84.1	69	85.2	106	84.8	.871
More advanced	7	15.9	12	14.8	19	15.2	
Clinical N stage							
0	9	20.5	20	24.7	29	23.2	.820
1	5	11.4	6	7.4	11	8.8	
2	29	65.9	54	66.7	83	66.4	
3	1	2.3	1	1.2	2	1.6	
Survival status							
Dead	34	77.3	44	54.3	78	62.4	.012
Alive	10	22.7	37	45.7	47	37.6	
Cause of death							
Distant metastasis	27	79.4	12	27.3	39	50.0	<.01
Reginal recurrence	1	2.9	2	4.5	3	3.8	
Local recurrence	0	0	12	27.3	12	15.4	
Others^∗^	6	17.7	18	40.9	24	30.8	
Surgical margin, mm							
≥5			12	14.8			
1–5			41	50.6			
<1			28	34.6			

*P* -value by *χ*^2^ test. CCI = Charlson Comorbidity Index, RMT = retromolar trigone.

∗ Including pneumonia, complication of adjuvant therapy, and other cancer related death.

Figure 1 presents the Kaplan–Meier curves of the 2 different treatment modalities based on whether patients were treated with or without surgery. These results exhibit significant differences between the 2 groups (*P* = .0001). Furthermore, Figure 2 presents the Kaplan–Meier curves for the 4 different treatment modalities based on surgery + CCRT, IC + surgery + CCRT, IC + CCRT, and CCRT alone. These results show that patients who received treatment modalities including surgery exhibited better survival than those who received treatment modalities without surgery (*P* = .0004).

**Figure 1:** Kaplan–Meier curves of 2 different treatment modalities based on whether patients underwent surgery.

**Figure 2:** Kaplan–Meier curves of patients treated with the 4 different treatment modalities. The 4 treatment groups are surgery + CCRT, IC + surgery + CCRT, IC + CCRT, and CCRT alone. CCRT = concurrent chemoradiation therapy, IC = induction chemotherapy, RT = radiotherapy, S = surgery.

Table 3 presents the survival time of patients treated with four different treatment modalities based on surgery + CCRT, IC + surgery + CCRT, IC + CCRT, and CCRT alone. These results show that the IC + surgery + CCRT group had the best survival outcome, with a mean OS time of 55.188 months.

**Table 3:** Survival of patients treated using the four different treatment modalities.

Treatment modalities	Mean, mo	SE	95% CIfor the mean	Median, mo	95% CI for the median
S + CCRT (n = 36)	47.989	6.345	35.554 to 60.425	43.64	18.590 to 93.020
IC + S + CCRT (n = 45)	55.188	7.101	41.270 to 69.105	51.05	21.250 to 109.840
IC + CCRT (n = 24)	27.061	5.061	17.143 to 36.980	12.46	7.900 to 57.970
CCRT only (n = 20)	20.537	4.865	11.002 to 30.073	7.44	5.080 to 24.430
Overall (n = 125)	43.749	3.916	36.074 to 51.425	25.18	18.590 to 109.840

CCRT = concurrent chemoradiation, IC = induction chemotherapy, RT = radiotherapy, S = surgery.

Table 4 presents the model contains treatment modalities based on whether patients were treated with or without surgery, tumor involving masticator space only, age at tumor was diagnosed whether >65 years’ old, CCI score was evaluated whether >4, tumor sites, and the surgical margin. In multivariate analysis, treatment modalities including surgery were shown as a sole indicator for achieving a better OS, and tumors primary located on tongue and hard palate resulted in poor prognosis.

**Table 4:** Multivariate analysis of clinical and pathological for overall survival.

Variable	Hazard ratio	Standard error	*P*	95% Confidence interval
Operation (yes vs no)	0.3705	0.2597	**.0001**	0.2227–0.6165
Tumor involving masticator space only (yes vs no)	1.2833	0.3614	.4901	0.6319–2.6062
Age at diagnosed ≧65	1.1901	0.3062	.5698	0.6530–2.1690
CCI score ≧4	0.9205	0.2593	.7494	0.5537–1.5302
Anatomic sites				
Alveolar ridge	1.0481	0.3224	.8842	0.5571–1.9718
Anterior tongue	5.1596	0.5599	**.0034**	1.7218–15.4614
Buccal mucosa	1			
Hard palate	2.0129	0.344	**.042**	1.0256–3.9505
Floor of mouth	0	186.7812	.951	1.0505–10.0947
Retromolar trigone	0.7489	0.4029	.4729	0.3400–1.6495
Mucosa of the lip	7.1427	1.0379	.0582	0.9341–54.6200
Surgical margin, mm				
≥5	0.5388	0.5481	.2591	0.1840–1.5773
1–5	1			
<1	1.4378	0.3272	.2672	0.7571–2.7305

CCI = Charlson Comorbidity Index.

## 4 Discussion

From 2012 to 2018, surgery was not the primary treatment for T4b OSCC, according to the NCCN guidelines. Obviously, the 2018 NCCN guidelines recommended that the preferred treatment modalities for very advanced OSCC (T4b) be clinical trials, systemic therapies, and radiotherapy based on the patient's performance status.^[2]^ In the present study, treatment modalities including surgery led to a better survival outcome than nonsurgical treatment modalities, despite that no significant differences were observed in the comorbidities of T4b OSCC patients between each treatment modality group.

Presently, published studies that discuss the treatment outcomes of patients with T4b OSCC are scarce. Baddour et al reported the outcomes of 25 patients diagnosed with T4b OSCC who underwent primary surgery. The OS rate beyond 24 months was 44%, and the patients who received postoperative adjuvant therapy had better survival outcomes than those who did not.^[9]^ Compared with our study, the OS rate was 63% in the first 24 months among T4b OSCC patients who received primary surgical treatment and only 39% in those who received nonsurgical treatment. Pillaia et al also compared the findings between 96 patients with T4a buccal OSCC and 181 patients with T4b who underwent primary surgical treatment. They reported that the survival rates after 2 years were 64% and 58% for T4a and T4b, respectively.^[10]^ Moreover, no significant survival difference was observed between the two groups according to a multivariate analysis, and extracapsular spread, lateral pterygoid muscle involvement, and default adjuvant treatment were independent predictors of outcome in patients with T4b. According to their conclusion, they proposed that primary surgical treatment followed by adjuvant treatment for select patients with T4b OSCC was feasible. Moreover, they recommended the need to update the OSCC staging system.^[10]^ Fang et al also reported the importance of multi-treatment modality for very advanced OSCC.^[7]^ In their study, they reported that 65 patients with T4b OSCC received a radical dose of intensity-modulated radiotherapy and that 33 patients were then treated with subsequent radical resection, whereas 32 patients were treated with adjuvant chemotherapy or observation. The 3-year OS rate was 75.1% in subsequent radical resection group compared with 47.7% in the nonsurgery group.^[7]^

Liao et al^[11]^ reported on the largest cohort of patients with T4b OSCC to date, and all patient data were available from the Taiwan Cancer Registry Database. Their study reported that, of all 492 patients with T4b OSCC, approximately two-thirds had received primary surgical treatment and that the cN0-2 classification represented a good prognosis. The 5-year OS rate in the primary surgical treatment group was 43% compared with 27% in the nonprimary surgical treatment group. The results were in agreement with those of our study. The patients who initially received nonsurgical treatment can be treated with surgery in order to achieve good outcomes. Although their study was reported in a larger database, one limitation cannot be ignored. Some differences in treatment discipline exist among various hospitals, and thus, the survival among patients at various hospitals could also be different. Compared with our study, all patients received treatment from the same head and neck surgery team, the same hematological team, and the same radiation oncology team, so that all complied with the same treatment protocols.

Performing surgery on a tumor located in the masticator space is challenging. This might be the main reason why clinicians are reluctant to choose primary surgical treatment for patients withT4b OSCC.^[4]^ When the tumor invades the masticator space, the patients’ maximal mouth opening could be restricted, and clinical assessment of tumor extension would be very difficult. The masticator space consists of multiple intertwined soft tissue structures, including the temporalis muscle, masseter muscle, medial and lateral pterygoid muscles, inferior alveolar nerve, pterygoid venous plexus, and internal maxillary vessels.^[3]^ All these soft tissue structures cause limitations to the preoperative determination of tumor invasion by MRI or CT. Moreover, it would be difficult to assess tumor invasion if intraoperative bleeding from the pterygoid venous plexus or internal maxillary vessels occurred.^[3,4]^ All these factors contribute to achieving negative margins in T4b OSCC, which is a very arduous process and is presumed to be the major reason why surgical treatment is still not the mainstay treatment for patients with T4b OSCC according to the NCCN guideline.^[2]^

Furthermore, to investigate suitable patients with T4b OSCC who were candidates for primary surgical treatment, Liao et al demonstrated that those patients with T4b OSCC with infra-notch tumor involvement who received primary surgical treatment exhibited significantly higher local control, neck control, disease-free survival, and OS rates compared with those with tumor supra-notch spread.^[5]^ Trivedi et al also reported a compartmental approach to remove total contents within the masticator space using an *en bloc* concept. The authors reported that this approach was the most feasible method that could achieve radical resection and that the 30 patients who received this treatment had good functional and acceptable esthetic results.^[3,12]^

Our study has several drawbacks. First, the data used in our study were collected from a single medical center in Taiwan, and the individuals in a single district may share numerous cultural and geographical features. Second, the sample size of patients with T4b limited the capacity for further stratified analysis. Finally, the present study was retrospective in nature, and significant biases may have affected the selection of controls.

## 5 Conclusions

In conclusion, to date, the published studies were limited, and various treatment methods have been reported. However, in the present study, patients with T4b OSCC who were treated with primary surgery had a better OS rate than those who received nonsurgical treatment. In the future, it will be necessary for clinicians worldwide to report the treatment outcomes of patients with T4b OSCC based on the common criteria.

## Acknowledgments

The authors thank Enago (www.enago.com) for the English language review. This research did not receive any specific grant from funding agencies in the public, commercial, or not-for-profit sectors.

## Author contributions

**Conceptualization:** Nan Chin Lin.

**Data curation:** Nan Chin Lin.

**Supervision:** Jui Ting Hsu.

**Writing – original draft:** Nan Chin Lin.

**Writing – review & editing:** Kuo Yang Tsai, Michael Chen.
